# PYRROLO[1,2-*b*][1,2,5]BENZOTHIADIAZEPINES (PBTDs) induce apoptosis in K562 cells

**DOI:** 10.1186/1471-2407-7-207

**Published:** 2007-11-09

**Authors:** Gabriella Marfe, Carla Di Stefano, Romano Silvestri, Elisabetta Abruzzese, Gianfranco Catalano, Livia Di Renzo, Giuseppe Filomeni, Ezio Giorda, Giuseppe La Regina, Emanuela Morgante, Maria Rosa Ciriolo, Matteo Antonio Russo, Sergio Amadori, Paola Sinibaldi-Salimei

**Affiliations:** 1 Department of Experimental Medicine and Biochemical Sciences, University of Rome "Tor Vergata", Rome, Italy; 2 Dipartimento di Studi Farmaceutici, University of Rome "La Sapienza", Rome, Italy; 3 Department of Haematology, University of Rome "Tor Vergata", Rome, Italy; 4 Department of Biology, University of Rome "Tor Vergata", Rome, Italy; 5 Research Center Ospedale Bambino Gesù, Rome, Italy; 6 Department of Experimental Medicine, University of Rome "La Sapienza", Rome, Italy; 7 IRCCS San Raffaele Pisana, Rome, Italy

## Abstract

**Background:**

The objective of this study was to gain insight into the molecular mechanism of induced cell death (apoptosis) by PYRROLO [1,2-*b*][1,2,5]BENZOTHIADIAZEPINES (PBTDs) series compounds, using human (K562) cells as a model.

**Methods:**

We focused our attention on some members of the PBTDs family to test their potential apoptotic activity in K562 cells. Important apoptotic activity was demonstrated, as evidenced by the concentration and percentage of cell death quantified by measuring PI-uptake by flow cytometry, and DNA fragmentation analyzed by agarose gel electrophoresis, generating a characteristic ladder pattern of discontinuous DNA fragments. The expression of Bcl-2 family was tested using western blotting and transfection method.

**Results:**

PBTDs-mediated suppression of K562 cell proliferation was induced by apoptosis characterized by the appearance of DNA fragmentation and was associated with the poly(ADP-ribose)polymerase (PARP) cleavage. PBTD-1 and -3 treatment resulted in caspase-3 activation through down-regulation of Bcl-2 and up-regulation of Bax. Furthermore, we used K562/vector and K562/bcl-2 cells, which were generated by transfection of the cDNA of the Bcl-2 gene. As compared with K562/vector, K562/Bcl-2 cells exhibited a 4-fold greater expression of Bcl-2. Treatment with 10 μM PBTD-1 and -3 for 24 h produced morphological features of apoptosis and DNA fragmentation in K562/vector cells, respectively. In contrast, PBTD-1 and -3-induced caspase-3 activation and apoptosis were inhibited in K562/Bcl-2. Furthermore, Bcl-2 overexpressing cells exhibited less cytocrome c release during PBTDs-induced apoptosis.

**Conclusion:**

These results indicate that PBTDs effectively induce apoptosis of K562 leukemia cells through the activation of caspase cascades. In addition, these findings indicate that Bcl-2 inhibits PBTD-1 and -3 induced-apoptosis via a mechanism that interferes with cytocrome c release, and the activity of caspase-3, which is involved in the execution of apoptosis.

## Background

The understanding of signals and pathways that regulate cell proliferation and apoptosis is crucial in searching devices capable diseases such as cancer. In fact, a raised threshold for apoptosis represents a central step in tumorigenesis, and tumors that possess alterations of the cell death signalling system are often resistant to chemiotherapy [1,2]. The evasion of apoptosis in response to death signals is achieved by malignant cell using set of mutations that inactive pro-apoptotic proteins or up-regulate anti-apoptotic protein [3].

Chronic myeloid leukaemia is an hematopoietic stem cell cancer cytologically characterized by the Philadelphia chromosome, which results from reciprocal translocation between chromosome 9 and chromosome 22 [4,5]. This mutation leads to the formation of the chimeric fusion protein Bcr/Abl, which manifests an uncontrolled tyrosine kinase activity. The expression of Bcr-Abl also contributes to confer apoptosis resistence after growth factors withdrawal or DNA damage. The ability to escape the normal death program provides a huge proliferative advantage and represents, especially during the accelerated or blast phase of disease, an obstacle to the successful treatment of this pathology, even when employing the new chemotherapic agent Imatinib [6-9]. In fact, Bcr-Abl kinase stimulates a variety of downstream survival pathways, including the mitogen-activated protein kinase cascade, Akt, the signal transducers and activators of transcription. Activation of these pathways in Bcr-Abl positive cells results in increased expression of several anti-apoptotic proteins, such Bcl-xl and Bcl-2, which block the release of cytocrome c from mithocondria, resulting in inactivation of caspases [10,11].

Two important groups of proteins involved in apoptotic cell death are the members of the Bcl-2 family [12] and a class of cysteine proteases known as caspases [13]. The Bcl-2 family can be classified into two functionally distinct groups: antiapoptotic proteins and pro-apoptotic proteins. Bcl-2, an antiapoptotic protein, is known for regulating apoptotic pathways and protecting against cell death. Bax, a pro-apoptotic protein of that family, is expressed abundantly and selectively during apoptosis and promotes cell death. Increasing the ratio of Bcl-2 to Bax has commonly been used to determine the induction of apoptosis in several tissues [14]. The caspases are aspartate-specific cysteine proteases that have emerged as the central executioner of apoptosis. Primary mechanism of apoptosis [13,15] goes through caspase-3 activation, which can be activated through cytosolic release of cytochrome c by Bax protein [16].

In the present study, we show that PBTDs suppresses proliferation of K562 cancer cells by causing apoptosis together with induction of proapoptotic Bcl-2 family members Bax and down-regulation of antiapoptotic proteins Bcl-2 and Bcl-xL, therefore leading to activation of caspases. In addition, overexpression of Bcl-2 inhibits PBTD-1 and -3 induced-apoptosis, which prevents the accumulation of cytocrome c in the cytosol, thereby preserving the caspase-3 in the inactive zymogen state and blocking molecular cascade of apoptosis.

## Methods

### Chemistry

Pyrrolo [1,2-*b*][1,2,5]benzothiadiazepines 5,5-dioxide (PBTDs) were developed in search for novel non-nucleoside anti-AIDS agents because they were discovered as potent inhibitors of the HIV-1 reverse transcriptase of HIV-1 [17]. In 2001 some pyrrolo[1,5]benzoxazepines were reported to induce apoptosis in CML cells by bypassing the apoptotic suppressor activity of the Bcr-Abl protein [16]. Taking into account these findings we selected some PBTD derivatives (compounds 1–3) having structural elements we thought crucial for the modulation of the apoptotic activity: (i) a benzofused heterocyclic ring; (ii) a sulfone group; (iii) a short side chain bearing COOH or COOR functions; (iv) an aroyl group at position 10 (Figure 1).

**Figure 1:** Molecular structures of PBTDs.

### Cells and Culture Conditions

The list and biological characteristics of long-tern cultured leukaemia cells that have been previously described and used in the present study, is illustrated in Table 1[18].

**Table 1:** Origin and biological characteristics of long-term cultured haematopoietic malignant cell lines used

No.	Line	Origin
1	K562	CML patient in blast crisis
2	HL- 60/M-	Promyelocitic human leukemia
3	U937	Promyelocitic human leukemia
4	Jurkat	acute T cell leukemia
5	IM-resistant K562	IM-resistant CML patient in blast crisis*

Resistant clones (IM-R-K562) are a gift from Carlo Gambacorti-Passerini (National Cancer Institute, Milan, Italy) (Morotti et al., 2006).

Cell lines were grown in suspension in RPMI 1640 medium supplemented with 10% (v/v) heated-inactivated fetal bovine serum (FbS) 100 U ml-1 of penicillin and 100 μg of streptomycin ml-1. For treatment with compounds 1, 3, exponential growing the different cells lines were collected and resuspended in fresh culture medium. Resistant clones (IM-R-K562) are a gift from Carlo Gambacorti-Passerini (National Cancer Institute, Milan, Italy) [19] and have been established by continuous exposure to imatinib as described [18]. No Bcr-Abl amplification nor Bcr-Abl point-mutations have been detected in this cell line (data not shown).

In the first series of experiments, K562 cells, were added in 25-cm culture flasks and incubated with different concentrations of in the range of 5, 10, and 15 μM for 24 hrs at 37°C. Briefly, then the cells maintained in RPMI 1640 medium supplemented for 3 hrs at 37°C. Furthermore, K562, HL60, Jurkatt, U937 and IM-R-K562 cells were treated PBTD-1 and-3 were incubated at the concentration 10 μM for 8, 16 and 24 hrs.

K562 cells stably transfected with an eukaryotic expression vector CMV/Bcl-2 (K562/Bcl-2) or control CMV/vector (K562/vector) vector.

### Assessment of cell viability

After exposure to PBTD-1 and -3, cell viability was assessed by propidium iodide (PI) exclusion. Cells (0.5 × 10^6^) were re-suspended in PBS and 50 μg/ml PI prior to flow cytometric analysis (FACScan; Becton Dickinson, Oxford, UK).

### DNA fragmentation assay

Briefly, cells were washed twice with phosphate-buffered saline (PBS) and lysed by addition of a hypotonic solution (1% NP-40 in 20 mM EDTA, 50 mM Tris-HCl pH 7.5). After centrifugation at 1600 × g for 5 min, the supernatant was collected and the extraction was repeated with the same lysis buffer. The supernatants was brought to 1% SDS and treated with RNase A (final concentration 5 mg/ml) for 2 h at 56°C followed by digestion with proteinase K (final concentration 2.5 mg/ml) at 45°C for at least 6 h. Before hydrolysis, a further cleaning of DNA was performed by phenol-chloroform extraction, followed by three successive ethanol precipitation in 2 M ammonium acetate. Pellets were dried for 30 min and resuspended in 200 μl Tris-EDTA pH 8.0 [20]. Aliquots of 20 μl containing 10 μg DNA were electrophoresed in 1.5% agarose gel.

### Protein extraction and Western blot analysis

Cells were homogenized directly into lysis buffer (50 mM HEPES, 150 mM NaCl, 1 mM EDTA, 1 mM EGTA, 10% glycerol, 1% Triton X-100, 1 mM phenylmethylsulfonyl fluoride, 1 μg/ml aprotinin, 0.5 mM sodium orthovanadate, and 20 mM sodium pyrophosphate). The lysates were clarified by centrifugation at 14,000 × 10 min. Protein concentrations were estimated by an assay (Bio-Rad) and boiled in Laemmli buffer (0.125 M Tris-HCl (pH 6.8), 4% SDS, 20% glycerol, 10% 2-mercaptoethanol, and 0.002% bromophenol blue) for 5 min before electrophoresis. Proteins were subjected to SDS-PAGE (12.5% polyacrylamide). After electrophoresis, proteins were transferred to nitrocellulose membranes (Immobilon, Millipore Corp., Bedford, MA); complete transfer was assessed using pre-stained protein standards (Bio-Rad, Hercules, CA). After blocking with Tris-buffered saline-BSA (25 mM Tris (pH7.4), 200 mM NaCl, and 5% BSA), the membrane was incubated with the primary antibodies. The following first antibodies, dissolved in 5% bovine serum albumin-TBST, were used: anti-Bax MAb (dilution 1:250) anti-BclXL MAb (dilution 1:250), anti-Bcl2 MAb (dilution 1:2,000), anti-poly(ADP-ribose) polymerase (PARP) (dilution 1:2000), anti-caspase-3 MAb (dilution 1:1,000) (all antibodies from Santa Cruz Biotechnology) and anti-β-actin MAb (dilution 1:7,500; Sigma). Membranes were then incubated with the horseradish peroxidase-conjugated secondary antibody (1:10,000) (at room temperature), and the reaction was detected with an enhanced chemiluminescence system (Amersham Life Science, Buckinghamshire, UK).

### Cytosolic protein extraction and cytochrome c immunoblot

Cytochrome c immunoblot was carried out using a modified protocol of Kluck et al. [21]. Cultured cells were treated with PBTD-1 and -3 in RPMI 1640 medium and then collected with lysis buffer (1 mM CaCl2, 1 mM MgCl2, 1% NP-40, 1 μg/ml leupeptin, 1 μg/ml aprotinin, 1 μM PMSF, and 100 μM NaVO4). After the lysis mixtures were incubated on ice for 20 mins, they were centrifuged at 14,000 rpm for 15 min. The supernatants were collected and total cytosolic proteins were quantitated by a Bradford spectrometer. About 80 μg protein was loaded in a 10% SDS-PAGE gel and transferred to polyvinylidene difluoride (PVDF) membrane at a constant current of 250 mA for 2 hours. The membrane was incubated with the primary cytochrome c polyclonal antibody (H-104, Santa Cruz) overnight at a dilution of 1:500. Horseradish peroxidaseconjugated anti-rabbit secondary antibody at a 1:1000 dilution was incubated with the membrane for another 1 hour at room temperature. The protein was detected with enhanced chemiluminescence for autoradiography

### Light and electron microscopy

The cells were fixed in 2.5% glutaraldhyde in 0.1 M PBS pH 7.3 and stored at 4 C. For processing the specimens were post-fixed for 1 h in 1.33% osmium tetroxide in 0.1 M PBS. Dehydratation and resin embedding were performed following a standard schedule. Semi-thin sections, 0.3 nm thick were cut, stained with Azur II and observed under a Nikon optical microscope. Ultra-thin sections, 70 nm thick were cut mounted on copper grid, stained with uranyl acetate and lead hydroxide and examined under a Philips CM-10 trasmission electron microscope at an accelerating voltage of 60 kV.

### Morphometry

The number of apoptotic cells was determined in 10 digital micrographs at magnification of 20. A total of 500 cells for each condition were studied. A Nikon Eclipse 1000 digital microscope equipped of Eclipse Net software has been used.

## Results

### PBTD-1 and -3 induced Apoptosis in cancer cells

To gain insights into the mechanism of PTBD-1 and -3 suppression of K562 cell proliferation, we determined its apoptotic effect by flow cytometry following staining with propidium iodide (Table 2, 3). Apoptosis induction by PBTD-1 and 3 was confirmed by analysis of DNA fragmentation and the results are shown in Figure 2A, 2B, 2C, 2D. The other cell lines were included in the analysis for direct comparison. Treatment of K562 cells with PBTDs resulted in a time-dependent manner and statistically significant increase of DNA fragmentation, compared to controls (figure 2). The effects of these agents were also examined in an imatinib mesylate-resistant CML cell line (IM-K562-R). Consistent with the results of cell survival assays, PTDBs treatment is able to cause DNA fragmentation in these cells (Figure 2D). All together, these results indicated that PBTDs-mediated inhibition of K562 cell proliferation was due to apoptosis induction.

**Table 2:** Percentage of the cell death was quantified measuring PI-uptake by flow cytometry. PBTD-3 10 μM.

Time hours	K562 % apop.	IM-Resistant K562 % apop	U937 % apop.	HL60 % apop	Jurkatt % apop
8	46	44	40	42	41
16	65	63	67	70	71
24	66	64	72	73	73

**Table 3:** Percentage of the cell death was quantified measuring PI-uptake by flow cytometry. PBTD-1 10 μM.

Time hours	K562 % apop.	IM-Resistant K562 % apop	U937 % apop.	HL60 % apop	Jurkatt % apop
8	34	32	38	39	39
16	60	59	65	66	67
24	64	63	66	68	69

**Figure 2:** Time-dependent DNA fragmentation. Cells were exposed to the indicated concentrations of synthetic compounds. Cells were harvested by centrifugation and DNA was extracted. The DNA fragments were separated on 1,8% agarose gel electrophoresis and visualized under ultraviolet. Cells were exposed to 10 μM PBTD-1 and PBTD-3 for 8,16, and 24 h.

Preliminary structure activity relationships (SARs) highlighted the crucial role of the ethoxycarbonyl fuction. In fact, independently from the 4-methylbenzoyl group at position 10 of the pyrrole [1,2-*b*][1,2,5]benzothiadiazepine ring, compounds 1 and 2 having an ethoxycarbonyl chain at position 11 were able to induce apoptosis. On the contrary, hydrolysis of the ester 1 to acid 2 led to a product deprived of apoptotic activity. Speculation about these findings suggests that arguably the acid 2 is less able to cross the cell membrane than the esters 1 and 3 one. In designing novel PBTDs as apotosis inductors it will be important to take in consideration the hydrophobic/hydrophilic balance as well as the ionic character of the molecule.

### Effect of PBTD-1 and -3 treatment on levels of Bcl-2 Family Proteins

We examined whether PBTDs induce cell death by modulating the expression of Bcl-2 family members, which ultimately determine the cell's response to apoptotic stimuli. The PBTD-1 and 3 treatment caused a rapid increase in the level of Bax protein. The PBTDs-mediated induction of Bax protein expression was evident as early as 8 hours after treatment and persisted along the experiment (24 hours after treatment).

The levels of antiapoptotic proteins Bcl-xL and Bcl-2 were initially increased after treatment with PBTDs (8 hours) but declined at 16- and 24-hour time points (Figure 3). Such results suggested that PBTDs-induced cell death might be regulated by Bcl-2 family proteins.

**Figure 3:** Immunoblotting for Bax, Bcl-xL, and Bcl-2 using lysates from K562 cells treated with 10 μM PBTD-1 and PBTD-3 for the indicated time periods. The blots were stripped and reprobed with anti-actin antibody to normalize for differences in protein loading. Immunoblotting for each protein was done at least twice using independently prepared lysates, and the results were comparable.

### Expression levels of bcl-2 overexpressed cells

In order to evaluate the functional role played by bcl-2 in preventing apoptosis induced by PBTDs, we first stably transfected K562 cells with a plasmid constitutively producing high levels of Bcl-2. Western Blot analysis revealed that K562/Bcl-2 cells exhibited a ~4-fold in bcl-2 expression compared with cell containg empty-vector (Figure 4A). In contrast, level of bax was equivalent in K562/Bcl-2 and K562/vector cells (Figure 4A).

**Figure 4:** A) Overexpression of Bcl-2 in K562 cells. Immunoblot analysis of cell lysate from control (K562/vector) or Bcl-2 transfected (K562/Bcl-2). The blot was probed with anti-Bcl-2 and anti-Bax. B) Fragmentation of genomic DNA in cells after treatment for 24 h with PBTD-1 and -3.

### Bcl-2 significantly prevents apoptosis induced by PBTDs

An important hallmark of apoptosis is the degradation of chromosomal DNA at internucleosomal linkages. We analyzed DNA fragmentation induced by in K562/Bcl-2 and K563/vector cells. Following agarose gel electrophoresis of K562/vector cells treated with 10 μM PBTDs for 24 h, a typical ladder pattern of internucleosomal fragmentation was observed (Figure 4B). In contrast, DNA fragmentation in K562/Bcl-2 was inhibited (Figure 4B).

### Involvement of Caspase-3 in PBTD-1 and -3-Induced Apoptosis

Our previous study demonstrated that the exposure to PBTDs for 24 h induces the activation of caspase-9 and 8 [22,23]. To determinate whether PBTDs-induced apoptosis was associated with the activation of caspase-3, we performed an immunoblotting that revealed cleavage of procaspase-3 after treatment with PBTD-1 and -3 for 8 to 24 hours (Figure 5A). In order to confirm the activation and execution of apoptosis by caspase-3, the cleavage of PARP (which is well accepted as one of the target proteins for caspase-3) was studied. As shown in Figure 5B, a PARP cleavage band was observed concomitantly with the occurrence of caspase-3 cleavage.

**Figure 5:** A. Immunoblotting for caspase-3 (full-length and cleaved intermediate) using lysates from K562 cells treated with 10 μM PBTD-1 and PBTD-3 for the indicated time periods. The blots were stripped and reprobed with anti-actin antibody to ensure equal protein loading. Immunoblotting for each protein was done at least twice using independently prepared lysates, and the results were comparable. B. PARP cleavage was also analyzed by immunoblotting under the same condition Data indicate 116 kDa PARP (upper bands) and 85 kDa apoptosis-related cleavage fragment (lower bands). C. K562/vector and K562/Bcl-2 cells were treated with PBTDs. Equal amounts of cell lysates were subjected to electrophoresis by western blot for caspase-3.

Furthermore, we determined the activity of caspase-3 in K562/bcl-2 and K562/vector cells. Caspase-3 is activared by proteolytic processing of the 32 KDa form into two smaller subunits. Activity of caspase-3 during PTBDs-induced apoptosis was measured by a decrease in pro-enzyme level using western blot analysis. As shown in Figure 5C, treatment resulted in a decrease in the level of caspase-3 in K562 cell control and K562/vector cells exposed 10 μM PTBDs for 24 h. In contrast, the levels of caspase-3 not significantly altered in PBTDs-treated K562/Bcl-2 (Figure 5C).

### PBTDs induce cytochrome c release in K562 cells

There is accumulating evidence that the mitochondria play an essential role in many forms of apoptosis by releasing apoptogenic factors, such as cytochrome c and apoptosis-inducing factor (AIF). Cytocrome c directly actives caspases by binding to Apaf-1 in presence of ATP [14]. To examine the release of cytocrome c in PBTDs-treated K562 cells K562/vector and K562/B, we conducted western blotting analysis. Importantly, the overexpression of anti-apoptotic Bcl-2 in k562 cells significantly blocked PBTDs-induced release of cytochrome c from mitochondria (Figure. 6A, 6B).

**Figure 6:** A. Cytochrome *c *release occurs between 8 and 24 after treatment. K562 cells were treated with both compounds and collected at each time point. The cytosolic and mitochondria-enriched fractions were prepared and western blot analyses were performed as described in Methods. B. K562/vector and K562/Bcl-2 were treated with PBTDs. The cytosolic and mitochondria-enriched fractions were prepared and western blot analyses were performed as described in Methods.

### Morphology

The light microscope analysis of semi-thin sections provided clear evidence of apoptosis in the K562 cells treated with PBTD-1 and -3. Figure 7 showed typical morphological apoptotic features consisting in: cytoplasmic vacuolization, patterns of chromatin condensation and micronuclei in K562 cells incubated with PBTD-3 compound.

**Figure 7:** A.-Most frequent nuclear apoptotic changes include: classical nuclear body formation with clumped chromatin and nuclear fragmentation. (× 9800); the bar represents 1 μm. (K562 treated with PBTD-3). B.-An other less frequent nuclear change is displayed in this picture: chromatin clumping and membrane complex fragmentation, likely due to the degradation of laminin fibers of nuclear dense lamina by caspase-3. Note the close association between nuclear membranes (paired cysternae) and clumped chromatin. (× 2000); the bar represents 3 μm.(K562 treated with PBTD-3). C.-A detail of the insert is shown. (× 9800); the bar represents 0,5 μm.

## Discussion

Increasing understanding of molecular bases of cancer has undoubtedly demonstrated that it is the inappropriate expression and activity of particular protein involved in intercellular and intracellular signalling networks that causes radical changes in cell behaviour, enabling prolonged cell survival and unlimited proliferative capacity.

Chronic myeloid leukaemia is paradigm of how an uncontrolled and perpetually switched on tyrosine kinase, like the fusion-protein Bcr-Abl, could turn normal cells into malignant ones [9]. Thus, considerable effort have been made for understanding the molecular mechanism underlying the transforming Bcr-Abl activity to possibly develop new therapeutic approaches, although several aspect are still obscure [6-11]. These considerations constituted the preamble of our study, which was at evaluating the possibility that PBTDs induce apoptosis in K562 cells.

PBTDs-induced apoptosis is mediated by caspase-3 activation, downregulation of Bcl-2 and Bcl-xL proteins and upregulation Bax protein. Furthermore, Bcl-2 overexpression blocks PBTDs-induced apoptosis in K562 cells by inhibition of caspase-3 activity.

Since the discovery of Bcl-2 as anti-apoptotic protein, several theories the Bcl-2 anti-apoptotic mechanism have been proposed [21,24,25]. The Bcl-2 anti-apoptotic function may explained by its ability to control several key steps of apoptosis signalling. Bcl-2 can form ion channels in biological membranes [26,27]. The ion channel activity of Bcl-2 may control apoptosis by influencing the permability of intracellular membranes and cytochrome c release from mitocondria [26,27]. The release of cytocrome c induces the activation of caspase-3 and DNA fragmentation. Our data showed that the release of cytochrome c from mithocondria in K562 cells preceded caspase activation by PBTDs. However, overexpression of Bcl-2 protein may rescue cells from apoptosis, blocking the release of cytocrome c from mitocondria and caspase-3 activation.

Thus, it seems that Bcl-2 family members play an important role in execution of PBDTs-induced cell death. Our findings suggest that these proteins are involved in the intracellular pathway leading to apoptotic death induced by these compounds. Taken together, the data indicate that the down-regulation of Bcl-2 and Bcl-xL and the upregulation of Bax could be responsible for PBTDs-induced apoptosis in K562 cells.

In summary, our studies demonstrate that PBTDs treatment of K562 cells induces cytochrome c release which activates pro-caspase-3 and DNA fragmentation. Moreover, expression of Bcl-2 inhibits PBTDs-induced apoptosis and prevents the release of cythocrome c from the mithocondria. Conventional cancer chemotherapeutic drugs indirectly induce cancer cell apoptosis, but more effective outcomes should be reached by direct activation of the apoptotic machinery. Accordingly, approaches of anticancer agents that cause down-regulation of antiapoptotic Bcl-2 family of proteins and/or up-regulation of proapoptotic Bcl-2 family of proteins should be carried out

## Conclusion

In view of accumulating evidence that PBTDs may be an important determinant of clinical response in leukaemia, further efforts to explore this therapeutic strategy appear warranted.

## Competing interests

The author(s) declare that they have no competing interests.

Patent application of PYRROLO[1,2-*b*][1,2,5]BENZOTHIADIAZEPINES (PBTDs): N. RM2005A000416, 3 August 2005;

Patent application N° PCT/IT2006/000401(International Pubblication Number WO 2007/015280 A1

## Authors' contributions

GM, CD, RS, GF, GL, EM participated in the design of study, and carried out coordinated the study. EA, GC, LD, EG, MRC. MAR, SA, PSS participated analysis and interpretation of data. EA and CD participated in the design of study and helped to draft the manuscript. GM conceived the study and participated in the design of study, analysis and interpretation of data, drafting the article and final approval of this version. All authors read and approved the final manuscript

## Pre-publication history

The pre-publication history for this paper can be accessed here:



## Supplementary Material

Additional file 1 Involvement of Caspases in PBTD-1 and -3-Induced Apoptosis. The expression of Bcr-Abl in bcl-2 overespressed cells. The data represent the involvement of caspases in agents-induced apoptosis and the role of Bcr-Abl in this process. Click here for file

Additional file 2 Immunoblotting for caspase-9 and caspase-8. Involvement of Caspases in PBTD-1 and -3-Induced Apoptosis. Click here for file

Additional file 3 Immunoblotting for Bcr-Abl protein. The expression of Bcr-Abl in bcl-2 overespressed cells Click here for file
